This article has been retracted.

# Role of MiR-27a-3p in Intervertebral Disc Degeneration through Targeting RASSF5 via MST1/LATS1 and RAS/RAC1 Signaling Pathway

**DOI:** 10.1155/2022/4457673

**Published:** 2022-03-07

**Authors:** Chao Yuan, Jing Zhou, Lei Zhou, Liran Wang, Yong Pan

**Affiliations:** Department of Orthopedics, Xinqiao Hospital, Army Medical University, Chongqing 400037, China

## Abstract

**Background:**

The apoptosis of nucleus pulposus (NP) cells reduces the number of nucleus pulposus cells in intervertebral disc tissue, resulting in intervertebral disc degeneration (IDD). MicroRNAs (miRNAs) play an important regulatory role in abnormal cell proliferation and apoptosis.

**Methods:**

The miR-27a-3p expressions in degenerative NP tissue and cells were measured via qPCR. The impacts of miR-27a-3p on the proliferation and apoptosis of human NP cells were evaluated by flow cytometry assays, MTT assays, and western blot analyses. In addition, target scan and luciferase reporter assay were applied to confirm that RASSF5 was directly binding to miR-27a-3p. Western blot was applied to assess the relationship between miR-27a-3p, RASSF5 and MST1/LATS1, and RAS/RAC1 signaling pathway.

**Results:**

MiR-27a-3p was downregulated in degenerative NP tissues and cells by comparison with the control group. MiR-27a-3p overexpression enhanced cell proliferation and suppressed apoptosis of NP cells, while the above factors showed an opposite tendency after in the miR-27a-3p inhibitor group. The western blot experiment similarly suggested mir-27a-3p apparently downregulated apoptosis-related proteins (Bax and caspase-3) and upregulated antiapoptotic proteins (Bcl-2). In addition, RASSF5 was confirmed to be directly regulated by miR-27a-3p using the luciferase reporter assay. Overexpressed RASSF5 could reverse the effects caused by miR-27a-3p mimic. Finally, miR-27a-3p could downregulate RASSF5 and affected the MST1/LATS1 and RAS/RAC1 pathway.

**Conclusion:**

MiR-27a-3p may target RASSF5 and enhance cell proliferation and imped cell apoptosis of the nucleus pulposus cells via the MST1/LATS1 and RAS/RAC1 pathway, lessening the degeneration of intervertebral discs.

## 1. Introduction

Intervertebral disc degeneration (IDD) plays a cardinal role in the progress of low back pain (LBP) [1]. About 70% of people are deeply affected by LBP which is considered as “the mystery of medical care in the 20th century” [2]. The number of IDD patients is increasing, which will lead to tremendous economic and healthy pressure on patients. The apoptosis of nucleus pulposus (NP) cells was reported to be one essential factor of the underlying mechanism of IDD [3]. The degeneration is mainly characterized by abundant NP cell apoptosis.

MicroRNA (miRNA) is a noncoding RNA molecule composed of 20 to 25 nucleotides, which is related to the regulation of cell growth, apoptosis, and migration through inducing or inhibiting of the translation of target genes [4]. A lot of microRNAs have been found to regulate the apoptosis of NP cells by binding to the 3'-UTR region of the target gene [5]. For instance, miR-150 [6], miR-15a [7], and miR-640 [8] have been proved to be related to the apoptosis of NP cells.

Many studies have reported RASSF5 was involved in a series of biological activities, especially related to cell proliferation and apoptosis. For instance, RASSF5 has been found to be regulated negatively by miR-532-5p to reduce alleviate IDD [9]. Xu et al. suggested RASSF5 enhanced cells apoptosis and suppressed proliferation in osteosarcoma [10]. According to the prediction of the TargetScan, RASSF5 was considered to be regulated by miR-27a-3p. According to Zhou et al.'s [11] study, miR-27a-3p can enhance cell proliferation in gastric cancer through downregulating the BTG2 expression. MiR-27a-3p was reported to enhance cell proliferation in lung cancer through targeting SLC7A11 [12].

Consequently, the purpose of present research was to study the functional role of miR-27a-3p in IDD and tried to verify it might impede NP cells apoptosis to inhibit IDD progression via targeting RASSF5.

## 2. Methods

### 2.1. Tissue Samples

According to MRI, twenty-three pairs of patients with scoliosis(grade II) and IDD(grade IV) were obtained from March 2017 and May 2019 and divided into control and disease groups (*n* = 23, average 24.9, range 18–26). Pfirrmann classification was adopted to grade the degree of disc degeneration. The protocols were approved by the agency, and the consents to use their tissues for scientific research were all signed by patients.

### 2.2. Cell Culture and Transfection

First of all, the sample tissue was washed cleanly using PBS, and the NP tissues were segregated by a stereotaxic microscope and trimmed into pieces. NP tissues were digested by incubation with 0.25 mg/mL type II collagenase (Corning, USA) for 6 hours at 37°C. The digest was filtered and centrifuged, and then supernatant was discarded. After inoculating the cells into the culture dish, cells were maintained in DMEM/F12 medium consisting of 15% foetal bovine serum (Corning, USA) and 1% penicillin-streptomycin (Corning, USA) for 3 weeks at 37°C and 5% CO_2_. The follow-up experiment was carried out with the third generation cells. The culture medium should be renewed once every three days. Overexpression or knockdown of miR-27a-3p was simulated by miR-27a-3p mimic or inhibitor which was purchased from GenePharma. NP cells were transfected with miR-27a-3p mimic/inhibitor, RASSF5, or empty vector into by Lipofectamine 2000 reagent (Thermo Fisher Scientific, USA).

### 2.3. RNA Isolation and Quantitative Real-Time PCR (qPCR)

The total RNA was extracted by TRIzol reagent (Beyotime Biotechnology, China). Subsequently, a nanodrop ultraviolet spectrometer (Thermo, USA) was applied to detect RNA concentration and purity. RNA was diluted with nuclease-free water and stored at −80°C for the next experiment. After RNA concentration determination, PrimeScript RT-polymerase (Takara, Japan) was applied to turning RNA into cDNA. The levels of the mRNAs of interest were determined by SYBR Green Premix (Takara, Japan). The primers sequences were synthesized by TsingKe (Shanghai, China). The 2^−ΔΔCT^ method was adopted to calculate miR-27a-3p expression, and the experiment was conducted three times.

### 2.4. MTT Assay

The MTT assay was adopted to detect the NP cell viability. About 2 × 10^3^ cells in each well were added into 96-well plates, which were incubated in 20 mL MTT at 37°C, subsequently. The microplate spectrophotometer was adopted to determine the absorbancy at 570 nm by at 12, 24, and 48 hours.

### 2.5. Flow Cytometry Assay

In order to measure apoptotic NP cells, FITC Annexin V/PI (BD Biosciences, CA) was adopted to dye cells. The cells, which were transfected with miR-27a-3p mimic/inhibitor for 48 h, were washed three times using PBS, and then binding buffer (10 mM HEPES/NaOH, pH 7.4; 140 mM NaCl; 2.5 mM CaCl_2_) was applied to resuspend these cells. Annexin V solution and PI were added to these cells. Subsequently, flow cytometry was adopted to detect the fluorescence intensity within 1 h.

### 2.6. Western Blot

Protein was abstracted by RIPA lysis buffer, and the concentration was analyzed using a BCA assay kit (Invitrogen, USA). Proteins were isolated using 10% SDS-PAGE gel electrophoresis. Subsequently, proteins were transferred to PVDF membrane (Corning, USA) which was blocked using the mixture consisting of 5% milk and PBST for 2 h at 25°C. After that, first antibodies with appropriate dilutions were used to incubate these membranes overnight at 37°C. The membrane was washed using TBST and incubated by secondary antibodies. The protein bands were imaged by the ECL immunoblotting kit (Tsingke, China). ImageJ Pro Plus software (Media Cybernetics, USA) was applied to measure each of protein bands and then was standardized according to its corresponding *β*-actin band.

### 2.7. Luciferase Reporter Assay

To create wild-type luciferase reporter vectors named wt-RASSF5 and the mutant reporter named mut-RASSF5, we inserted the wild-type or mutant miR-27a-3p binding site in 3'UTR of RASSF5 into the pGL3 vector (Promega, USA). Cells were cotransfected with wt-RASSF5 3ʹUTR or mut-RASSF5 3ʹUTR and miR-27a-3p mimic by LipofectamineTM2000. Then, Dual-Luciferase Reporter Assay was adopted to detect luciferase activity after 48 h.

### 2.8. Statistical Analysis

SPSS 20.0 software was adopted to analyze all data. *T*-test and one-way ANOVA were conducted to figure out the difference between groups. *P* < 0.05 can be considered as that the difference between groups is significant. GraphPad Prism 8 software was applied to draw graphs.

## 3. Results

### 3.1. MiR-27a-3p mRNA Expression Was Downregulated in IDD Tissues and Cells

We firstly measured the relative expression of miR-27a-3p in degenerative NP tissue and cells using qPCR. MiR-27a-3p was lower expressed in degenerative NP tissues by comparison with the control group (Figure 1(a)). Furthermore, miR-27a-3p was lower expressed in degenerative NP cells by comparison with the control group (Figure 1(b)).

### 3.2. MiR-27a-3p Suppressed NP Cell Apoptosis and Promoted NP Cell Proliferation

RT-qPCR was applied to detect miR-27a-3p expression; after that, NP cells were transfected by miR-27a-3p mimic/inhibitor, and the result suggested that miR-27a-3p mimic obviously overexpressed miR-27a-3p, while miR-27a-3p inhibitor reduced miR-27a-3p expression (Figure 2(a)). MMT assay was adopted to examine cell proliferation. Cell proliferation in the miR-27a-3p mimic group was obviously raised, while miR-27a-3p inhibitors inhibited cell proliferation by comparison with the NC group (Figure 2(b)). Flow cytometry assay was performed to analyze NC cells apoptosis. As shown in Figure 2(c), apoptosis of NC cells in the miR-27a-3p mimic group was reduced, while miR-27a-3p inhibitors increased NP cell apoptosis. Furthermore, the Bcl-2 expression was raised, while Bax and caspase-3 were significantly decreased in the miR-27a-3p mimic group. Contrarily, expression of Bcl-2 was obviously lowered in comparison with the NC group, while Bax and caspase-3 were observably raised in the miR-27a-3p inhibit group (Figure 2(d)).

### 3.3. MiR-27a-3p Directly Regulated RASSF5

RASSF5 was predicted to be regulated by miR-27a-3p using TargetScan forecast (Figure 3(a)). In order to more directly prove that RASSF5 is regulated by miR-27a-3p, the luciferase reporter assays were conducted. Results suggested miR-27a-3p mimic decreased the luciferase activities of the wt-RASSF53ʹUTR, while it showed unconverted effects on the mut-RASSF5 3ʹUTR (Figure 3(b)). Consistently, the expression of RASSF5 reduced in the miR-27a-3p mimic group and raised in the miR-27a-3p inhibit group in NP cells (Figure 3(c)).

### 3.4. Overexpression of RASSF5 Attenuated the Promoting Effect of MiR-27a-3p on NP Cell Proliferation

In order to better understand the mechanism of miR-27a-3p on the occurrence and progress of IDD, miR-27a-3p mimic was cotransfected into NP cells with oe-RASSF5. As shown in Figure 4(a), miR-27a-3p overexpression raised NP cells proliferation, while RASSF5 overexpression decreased it. MiR-27a-3p overexpression significantly decreased the number of apoptosis cells, while it recovered in miR-27a-3p mimic + oe-RASSF5 group (Figures 4(b) and 4(c)). The protein expression of Bcl-2 was observably raised in the miR-27a-3p mimic group but reduced in the miR-27a-3p mimic + oe-RASSF5 group. Contrarily, protein expression of Bax and caspase-3 was observably reduced but raised in the miR-27a-3p mimic + oe-RASSF5 group (Figure 4(d)).

### 3.5. MiR-27a-3p Promoted NP Cell Proliferation and Inhibited Apoptosis through MST1/LATS1 and RAS/RAC1 Signaling Pathway

Results above revealed miR-27a-3p aggravated NP cells proliferation and repressed apoptosis by regulating RASSF5 directly. We investigated which signaling pathway is related to this biological process. Western blot assays were adopted to examine protein expression of p-MST1, p-LATS1, RAS, and RAC1. Results indicated that miR-27a-3p overexpression decreased expression of RASSF5, p-MST1, and p-LATS1 and overexpressed RASSF5 overturned the impact of miR-27a-3p mimic (Figure 5(a)). MiR-27a-3p overexpression significantly increased protein expression of RAS and RAC1 and overexpressed RASSF5 overturned the impact of miR-27a-3p mimic (Figure 5(b)).

## 4. Discussion

As we all know, IDD is the main cause of low back pain, and it is the worldwide common musculoskeletal disease. More and more evidence shows the miRNA is related to the prognosis and progress in a variety of cancers which might become the target of gene therapy in the future. MiR-150 was reported to bind to P2X7 to reduce the degeneration of intervertebral disc in rats via the NF-*κ*B pathway, leading to inhibit apoptosis of the NP cells [6]. MiR-133a has been found to directly target to MMP9, repressing progress of intervertebral disc degeneration by inhibiting type II collagen loss [13]. In the present research, the mir-27a-3p expression in degenerative NP tissue, and cell was obviously lower in comparison with the control group. A lot of reports showed that mir-27a-3p was higher expressed in a series of cancers and impede cell apoptosis [14–16]. Mir-27a-3p in glioma tissues was obviously expressed lower in comparison with the control group. Mir-27a-3p targeted to MXI1 to impede cells apoptosis [16]. The present research obtained similar result which indicated high expression of miR-27a-3p enhanced NP cell proliferation and inhibited cells apoptosis. The western blot experiment results were consistent. Mir-27a-3p increased the expression of antiapoptotic proteins of Bcl-2 and decreased the expression of apoptosis related proteins of Bax and caspase-3.

Through TargetScan, we predicted that RASSF5 was binding to miR-27a-3p. RASSF5 was proved as a downstream gene of miR-27a-3p through luciferase reporter assays. MiR-27a-3p overexpression obviously decreased the luciferase activities of wt-RASSF5 but showed unconverted effects on the mut-RASSF5. We measured the protein expression of RASSF5 after over/low expressed miR-27a-3p levels. Consistently, miR-27a-3p overexpression obviously reduced the expression of RASSF5, and miR-27a-3p inhibitor increased the expression of RASSF5 in NP cells. There have been some studies shown that RASSF5 is regulated by microRNAs such as miR-532-5p [9], miR-214 [17], and miR-486-5p [18] and plays a cardinal role in cell proliferation and apoptosis. According to the paper of Zhu miR-532-5p regulated RASSF5 negatively to inhibit cell apoptosis and reduce alleviate IDD [9]. Zhou et al. suggested that RASSF5 suppressed the proliferation and promotes apoptosis of osteosarcoma cells [10]. Because we found the miR-27a-3p enhanced NP cells proliferation, we further investigated whether RASSF5 is a downstream gene of mir-27a-3p. We confirmed this conjecture by MTT, flow cytometry, and western blot experiments, which suggested that overexpression of RASSF5 attenuated the effect of miR-27a-3p on NP cells.

According to the previous research, RASSF5 could involve in the MST1/LATS1 signaling pathway [19–21] and RAS/RAC1 signaling pathway [22, 23] which are crucial to cells proliferation and apoptosis. Consequently, we assumed miR-27a-3p might regulate the MST1/LATS1 and RAS/RAC1 signaling pathway in IDD by targeting RASSF5. Results indicated overexpressed miR-27a-3p observably decreased protein expression of RASSF5, p-MST1, and p-LATS1 and overexpressed RASSF5 showed the opposite effect on these proteins. Moreover, overexpressed miR-27a-3p observably raised protein expression of RAS and RAC1 and overexpressed RASSF5 showed the opposite effect on these proteins. The result revealed that the miR-27a-3p could affect NP cell proliferation apoptosis by targeting RASSF5 via MST1/LATS1 and RAS/RAC1signaling pathway in IDD.

## 5. Conclusion

Consequently, the present research indicated miR-27a-3p may target RASSF5 to enhance cell proliferation and imped cell apoptosis of the nucleus pulposus cells via the MST1/LATS1 and RAS/RAC1 pathway, lessening the degeneration of intervertebral discs.

## Figures and Tables

**Figure 1:** The miR-27a-3p expression in degenerative NP tissue and cell. (a) Low expression miR-27a-3p in degenerative NP tissues (*N* = 23). (b) Low expression of miR-27a-3p in degenerative NP cells. ^∗^*P* < 0.05.

**Figure 2:** Overexpressing miR-27a-3p impeded NP cells apoptosis and enhanced cell proliferation. (a) The expression of miR-27a-3p in NP cells. (b) Hindrance effect of miR-27a-3p inhibitor and promoting effect of miR-27a-3p mimic on NP cell proliferation. (c) Promoting effect of miR-27a-3p inhibitor and hindrance effect of miR-27a-3p mimic on cell apoptosis. (d) The expression of apoptosis-related proteins was measured via western blotting. ^∗^*P* < 0.05.

**Figure 3:** MiR-27a-3p downregulates the RASSF5 expression via binding its 3'UTR. (a) Diagrammatic sketch of the RASSF5 3'-UTR. (b) Inhibiting effect of miR-27a-3p mimic on luciferase activity of RASSF5-WT. (c) The effect of miR-27a-3p mimic/inhibitor on expression of RASSF5. ^∗^*P* < 0.05.

**Figure 4:** The effect of RASSF5 on NP cells proliferation and apoptosis regulated by miR-27a-3p. (a) oe-RASSF5 attenuated miR-27a-3p mimic promoting effect on NP cell proliferation. (b, c) oe-RASSF5 attenuated impact of miR-27a-3p mimic on NP cell apoptosis. (d) oe-RASSF5 attenuated impact of miR-27a-3p mimic on the expression of apoptosis-related proteins. ^∗^*P* < 0.05.

**Figure 5:** Impact of miR-27a-3p and RASSF5 overexpression on MST1/LATS1 and RAS/RAC1 signaling pathway. (a) Impact of miR-27a-3p and RASSF5 on the MST1/LATS1 signaling pathway. (b) Impact of miR-27a-3p and RASSF5 on the RAS/RAC1 signaling pathway. ^∗^*P* < 0.05.

## Data Availability

Data to support the findings of this study are available upon reasonable request from the corresponding author.
